# Inhibition of miR-421 Preserves Mitochondrial Function and Protects against Parkinson's Disease Pathogenesis via Pink1/Parkin-Dependent Mitophagy

This article has been retracted.

**DOI:** 10.1155/2022/5186252

**Published:** 2022-05-10

**Authors:** Xiaolin Dong, Xianghua He, Li Yang, Qingyun Li, Yanming Xu

**Affiliations:** ^1^Department of Neurology, West China Hospital, Sichuan University, Chengdu, China; ^2^Department of Neurology, The Affiliated YanAn Hospital of Kunming Medical University, Kunming, China

## Abstract

Mutations in PINK1 and Parkin are a major cause of Parkinson's disease (PD) pathogenesis. In addition, PINK1 and Parkin are two mitochondrial proteins that jointly contribute to mitochondrial homeostasis via mitophagy. Mitochondrial dysfunction is the most significant mechanism underlying PD pathogenesis. Thus, understanding the regulatory mechanism of PINK1 and Parkin expression is beneficial to the treatment of PD. In this study, we found that miR-421 expression was upregulated in mice treated with MPTP, as well as in SH-SY5Y cells treated with methyl-4-phenylpyridine (MPP+). Inhibition of miR-421 alleviated neurodegeneration in MPTP-treated mice and promoted mitophagy in MPP+-treated SH-SY5Y cells. Bioinformatics software predicted that Pink1 is a downstream target protein of miR-421. In addition, miR-421-induced Pink1 and Parkin inhibition negatively modulates mitophagy in MPP+-treated SH-SY5Y cells. In addition, our study confirmed that Pink1/Parkin is responsible for miR-421-regulated cell mitophagy. Overall, this study revealed that miR-421 regulates nerve cell mitophagy through the Pink1/Parkin pathway.

## 1. Introduction

Parkinson's disease (PD) is a disease associated with the loss of nigrostriatal dopaminergic neurons and is the second most common neurodegenerative disorder [1, 2]. Mitochondria play an important role in neuronal homeostasis and function [3]. Indeed, mitochondrial impairment is one of the most important hallmarks of PD, and the accumulation of damaged mitochondria has been reported as a major driving mechanism for PD [4, 5]. Moreover, studies have indicated that mitochondria could be potential targets for PD treatment [6, 7]. Mitophagy is a degradation process that clears damaged mitochondria and maintains mitochondrial function [8, 9]. A growing number of studies have demonstrated that mitophagy is involved in PD pathogenesis [10]. However, the mechanisms by which mitophagy regulates PD are not entirely clear.

The mitochondrial proteins, PINK1 and Parkin, are linked to heritable PD [11]. Moreover, abnormal expression of PINK1 and Parkin is thought to be a major cause of PD [12, 13]. Studies have demonstrated the involvement of PINK1 and Parkin in the mitophagy process. For instance, cadmium enhances mitophagy in PC cells via PINK1 and Parkin [14]. PINK1/parkin-mediated mitophagy is critical for neuroprotection [15].

microRNAs are small RNAs that regulate the transcription of target genes [16]. Altered expression of miRNA could be observed in PD, which suggests that miRNA functions as a critical regulatory factor in PD [17–19]. Indeed, miRNAs can be potential biomarkers and provide new insights into PD pathogenesis [20, 21]. The regulation of apoptosis and autophagy by miR-421 plays an important role in neuronal function [22, 23]. Notably, the involvement of miR-421 in mitochondrial regulation has been reported. In cardiac disease, miR-421 regulates mitochondrial fragmentation and cardiomyocyte apoptosis [24]. Oleanolic acid (OA) derivative-regulated miR-421 inhibits mitochondrial function in pancreatic cancer [25]. Meanwhile, miR-421 has been reported to increase neurotoxicity and promote cell death in Parkinson's disease models by directly targeting MEF2D [26]. Therefore, we hypothesized that miR-421 can aggravate neurotoxicity in Parkinson's disease models by affecting mitochondrial autophagy and carried out further exploration.

In the present study, we identified a novel regulatory mechanism of PINK1 and Parkin by miR-421. We show that inhibition of miR-421 upregulates PINK1 and Parkin, thereby promoting mitophagy and maintaining mitochondrial function in PD.

## 2. Materials and Methods

### 2.1. Cell Culture and Treatment

For SH-SY5Y and H293T (ATCC), the cell culture medium was DMEM containing 10% FBS (Gibco, 10099141) and 1% streptomycin/streptomycin sulfate (Gibco, 15140122), and the culture conditions were 37°C and a 5% CO_2_ incubator. Methyl-4-phenylpyridinium (MPP+) was used for PD cellular model establishment. The different concentrations (0 mM, 0.25 mM, 0.5 mM, and 1 mM) of MPP+ treated the cells for 24 h.

### 2.2. Cell Transfection

SH-SY5Y cells were inoculated into 6-well plates (1 × 10^6^ cells/well) and cultured at 37°C until 80% confluence before transfection. The miR-421 inhibitor and control miR-421 inhibitor were purchased from RiboBio. Small interfering RNA (siRNA) specifically targeting PINK1 (siPINK1, 5′-CCAAGCGCGTGTCTGACCC-3′) and the NC siRNA (siNC, 5′-ATGGGTCAGCACGTTCAGTTA-3′) were synthesized by GenePharma. They were transfected into SH-SY5Y cells. Transfection was conducted according to Lipofectamine 3000 (Invitrogen) instructions. After 48 h of transfection, the cells were treated with 0.5 mM MPP+ for 24 h.

### 2.3. Mitochondrial Isolation

The mitochondria were isolated with a mitochondrial extraction kit (Solarbio, SM0020). The cells were lysed with lysis buffer. The supernatant was centrifuged for 10 min at 12, 000*g* three times, and the mitochondrial precipitate was collected. The mitochondria were washed and resuspended in store buffer. The isolated mitochondrial fraction was used for MMP and LC3II/I protein level determination.

### 2.4. Cell Apoptosis Assay

SH-SY5Y indicator cells were collected after transfection. An Annexin V-FITC/PI double staining kit (Invitrogen) was used for the quantitative detection of apoptotic cells. Annexin V was added first, and then, PI solution was added. The mixture was incubated at room temperature in the dark for 15 minutes. The early and late apoptosis of the cells was examined by flow cytometry. Fluorescence signals of cells stained with FITC and PI were collected in the 620-nm and 525-nm emission channels, respectively.

### 2.5. Detection of ROS

The production of ROS was determined according to the instructions of the cellular ROS assay kit (Abcam, ab186029). SH-SY5Y cells and ROS deep red dye working solution were incubated at 37°C for 60 minutes. Changes in fluorescence intensity (Ex/m = 650/675 nm) were monitored by flow cytometry.

### 2.6. Mitochondrial Membrane Potential Measurement

The Δ*ψm* was analyzed by measuring the fluorescence intensity of cells stained with JC-1 dye (Abcam, ab141387). SH-SY5Y cells were trypsinized, washed with PBS buffer, and resuspended in DMEM. SH-SY5Y cells were incubated with JC-1 dye for 45 minutes, and the fluorescence intensity of the mixture was analyzed by flow cytometry after resuspending the cells in PBS buffer.

### 2.7. Quantitative Real-Time Polymerase Chain Reaction (RT-qPCR)

Total cellular RNA extracted from the cells and tissues was measured using TRIzol reagent (Beyotime, R0016). cDNA was synthesized with PrimeScript™ RT reagent Kit (Takara, RR037A). RT-qPCR was performed with SYBR qPCR Master Mix (Vazyme, Q311-02). miR-421, sense: TCAACAGACATTAATTGGGCG, antisense: CTCAACTGGTGTCGTGGAGTC. U6, sense: TTATGGGTCCTAGCCTGAC, antisense: CACTATTGCGGGTCTGC.

### 2.8. Western Blot Assay

Total proteins from tissues and cells were isolated by RIPA lysis buffer. The protein concentration was determined by BCA (Beyotime, P0012). Proteins (40 *μ*g per lane) were loaded in sodium dodecyl sulfate–polyacrylamide gel electrophoresis and then transferred onto polyvinylidene difluoride (PVDF) membranes. PDFV membranes were blocked with nonfat milk and incubated with primary antibodies against GAPDH (Abcam, ab9485), LC3 (Cell Signaling Technology, 2775), PINK1 (Abcam, ab23707), and Parkin (Abcam, ab233434). The primary antibody was incubated overnight at 4°C and combined with the secondary antibody (Abcam, ab205718).

### 2.9. Luciferase Assay

The relationship between miR-421 and PINK1 was detected by a luciferase reporter assay. The PINK1 3′UTR fragment was cloned into the pmirGLO vector (LMAI Bio, LM-1439), and the transferred fragment contained the predicted wild-type or mutant-binding sequence of miR-421. Then, SH-SY5Y cells were cotransfected with pmirGLO vectors and miR-421 mimics or NC mimics. After 48 h, the luciferase activity of the cells was detected with a double luciferase reporting kit (Beyotime, RG027).

### 2.10. Animals

The C57BL/6 mice were purchased from Kunming Medical University Animal Center. MPTP was intraperitoneally injected at 20 mg/kg/d for 14 consecutive days. The control group was intraperitoneally injected with an equal volume of normal saline, and the operation and precautions were the same. For miR-421 inhibitor treatment, MPTP-treated mice were injected with miR-421 inhibitor. Mice were randomly divided into the control group, MPTP group, NC inhibitor group, and miR-421 inhibitor group.

### 2.11. Immunohistochemistry

After anesthetization, the brains of the mice were removed, fixed in 4% formaldehyde fixative, and then dehydrated in gradient ethanol. The brain was paraffin-embedded and sectioned. Immunohistochemical analysis was performed with tyrosine hydroxylase (TH) polyclonal antibody (Abcam, ab112).

### 2.12. Statistical Analysis

The data are represented as the mean ± standard deviation (SD). Student *t* test was used for comparisons between two groups, and one-way of variance (ANOVA) was used for comparisons between multiple groups. Significance was accepted at *P* < 0.05.

## 3. Results

### 3.1. MiR-421 Is Highly Expressed in MPP+-Intoxicated SH-SY5Y Cells and Inhibits Mitophagy

Following the stimulation of SH-SY5Y cells with MPP+ (0 mM, 0.25 mM, 0.5 mM, and 1 mM) for 24 h, increased miR-421 levels could be observed according to the RT-qPCR results (Figure 1(a)). These results suggested that miR-421 may be involved in PD pathogenesis. To verify the function of miR-421 in a cellular model of PD, we first knocked down miR-421 by miR-421 inhibitor transfection. RT-qPCR results showed that the expression of miR-421 was significantly downregulated after transfection with miR-421 inhibitor, indicating that the transfection was successful (Figure 1(b)). We found that inhibition of miR-421 could attenuate the promotion of apoptosis by MPP+ in SH-SY5Y cells. Western blot detection of the expression of the apoptosis protein Bax showed that after the SH-SY5Y cells were treated with MPP+ (0.5 mM), Bax was significantly upregulated compared with that in the control group, but SH-SY5Y cells were first transfected with miR-421 inhibitor and then MPP+ after treatment. The expression of Bax in the MMP+ + miR-421 inhibitor group was decreased compared with that in the MMP+ + NC inhibitor group (Figure 1(c)). Flow cytometry detection of SH-SY5Y cell apoptosis also found that MPP+ can promote the apoptosis of SH-SY5Y cells, but transfection of miR-421 inhibitor can effectively alleviate the promoting effect of MPP+ on SH-SY5Y cell apoptosis; that is, compared with the MMP+ + NC inhibitor groups, the apoptosis of the MMP+ + miR-421 inhibitor group decreased (Figure 1(d)). It has been reported that mitophagy plays a significant role in PD pathogenesis and diagnosis [10, 27]. Here, we showed that the level of mitophagy decreased after MPP+ administration. Western blot test results showed that MPP+ treatment significantly reduced the expression of LC3II/I protein and inhibited the occurrence of SH-SY5Y cell autophagy, while transfection with miR-421 inhibitor reversed the inhibition of MPP+ on SH-SY5Y cell autophagy to a certain extent (Figure 1(e)). The increase in ROS levels and the decrease in mitochondrial membrane potential (*Δψ*m) in SH-SY5Y cells induced by MPP+ treatment were also reversed to some extent after the inhibition of miR-421 (Figures 1(f) and 1(g)).

### 3.2. MiR-421 Directly Targets PINK1 and Decreases the Expression of PINK1 and Parkin

It has been reported that miR-421 has a targeted binding site with PINK1 [24, 28]. We also predicted the targeted binding site between miR-421 and PINK1 through bioinformatics software and further confirmed the targeted binding relationship between miR-421 and PINK1 through a double luciferase gene reporter experiment (Figure 2(a)). Studies have demonstrated that the PINK1/Parkin pathway is responsible for mitophagy [29]. In our study, the results of Western blot detection showed that the expression levels of PINK1 and Parkin were downregulated after MPP+ treatment of SH-SY5Y cells, and the inhibition of miR-421 could restore the expression levels of PINK1 and Parkin to a certain extent; that is, compared with the MMP+ + NC inhibitor group, the expression levels of PINK1 and Parkin were upregulated in the MMP+ + miR-421 inhibitor group (Figure 2(b)).

### 3.3. MiR-421 Inhibits Cell Mitophagy via PINK1/Parkin in MMP-Treated SH-SY5Y Cells

To determine whether miR-421 inhibits cellular mitophagy through PINK1/Parkin, a miR-421 inhibitor was transfected or cotransfected with miR-421 inhibitor+siPINK1 before MPP+ treatment of SH-SY5Y cells. WB detection showed that transfection of the miR-421 inhibitor upregulated the expression of PINK1 and Parkin, but cotransfection of the miR-421 inhibitor+siPINK1 reversed the promotion effect of miR-421 inhibition on the expression of PINK1 and Parkin (Figure 3(a)). The expression of the apoptosis protein Bax was detected by Western blotting, and the expression was upregulated in the miR-421 inhibitor+siPINK1 group compared with the miR-421 inhibitor+con group (Figure 3(b)). Flow cytometry also showed increased apoptosis in the miR-421 inhibitor+siPINK1 group compared with the miR-421 inhibitor+con group (Figure 3(c)). Western blot test results showed that the inhibitory effect of MPP+ treatment on LC3II/I protein expression was weakened by the transfection of the miR-421 inhibitor, but this effect was reversed by the cotransfection of miR-421 inhibitor+siPINK1 (Figure 3(d)). Likewise, the increase in ROS levels and the decrease in mitochondrial membrane potential (*Δψ*m) in SH-SY5Y cells induced by MPP+ treatment were inhibited by transfection with the miR-421 inhibitor, but the above phenomenon was also reversed by cotransfection with miR-421 inhibitor+siPINK1; that is, ROS increased, and *Δψ*m decreased in the miR-421 inhibitor+siPINK1 group compared with in the miR-421 inhibitor+ con group (Figures 3(e)-(f)).

### 3.4. Inhibition of miR-421 Attenuates Neurodegeneration in Mice

We determined the role of miR-421 in MPTP-treated mice by treating PD mice with miR-421 inhibitor and control miR-421 inhibitor. First, RT–qPCR results showed that miR-421 expression was significantly upregulated in miR-421-treated brain tissues of PD mice, while miR-421 inhibitor injection reduced the expression of miR-421 in the brain tissues of PD mice (Figure 4(a)). Meanwhile, we found that the expression levels of PINK1 and Parkin were significantly downregulated in the brain tissues of MPTP-induced PD mice, while the expression levels of PINK1 and Parkin could be improved to a certain extent with the injection of the miR-421 inhibitor (Figure 4(b)). Finally, the expression changes of TH in mouse brain tissues were detected by immunohistochemistry, and the results showed that TH-positive cells were significantly reduced in MPTP-induced PD mice, while the inhibition of miR-421 reduced TH loss (Figure 4(c)).

## 4. Discussion

In this study, we demonstrated the role of miR-421 in regulating mitochondrial function through PD cell models and animal models. We found upregulation of miR-421 expression in both MPP+-treated SH-SY5Y cells and MPTP-treated mice. Inhibition of miR-421 attenuates neurodegeneration in MPTP-treated mice. MiR-421 suppression restrained cell apoptosis and facilitated mitophagy in MPP+-intoxicated SH-SY5Y cells, thereby maintaining mitochondrial function. Furthermore, we found that miR-421 could directly target PINK1, which is a mitochondrial protein involved in mitophagy modulation. miR-421 knockdown enhanced PINK1 and Parkin expression. Our results indicate that PINK1/parkin-mediated mitophagy was responsible for miR-421-regulated mitophagy in the progression of PD.

Mitochondrial dysfunction is one of the most significant hallmarks of PD [30]. In addition, mitochondria have been reported as potential therapeutic targets for PD. For instance, treatment with ursocholanic acid relieved PD by rescuing mitochondrial function [7]. Metformin alleviates PD phenotypes by modulating mitochondrial activity [31]. Mitophagy is a degradation process for maintaining mitochondrial quality and homeostasis [32]. Our results showed that in the MPP+-induced PD cell model, the expression of the autophagy-related protein LC3II/I was significantly decreased, the level of ROS in the cells increased, and the mitochondrial membrane potential (*Δψ*m) decreased, indicating that autophagy inhibition occurred in PD. This evidence suggests that mitochondrial autophagy-mediated mitochondrial dysfunction plays a key role in the pathogenesis of PD. Thus, it is necessary to discover potential targets for maintaining mitochondrial function.

MiRNAs are small noncoding RNAs that participate in a variety of cellular activities and play an important role in gene expression regulation [22]. The role of miRNAs in PD pathogenesis has been well characterized. Aberrant expression of miRNAs could be a biomarker for PD. For example, differential expression of miR-27a-3p is associated with early onset of PD [33]. Cressatti et al. indicated that the levels of miR-153 and miR-223 in saliva can be diagnostic biomarkers for PD [34]. Sun et al. showed that miR-190 is downregulated in a PD mouse model and alleviates neuronal damage and neuroinflammation [35]. miR-421 is a critical regulator of PD development [26]. In our study, we found that miR-421 expression was significantly upregulated in both PD cells and animal models. The mitochondrial protein PINK1 plays an important role in mitophagy [36]. The activity of PINK1 can be modulated by miRNAs [37]. At the same time, various studies indicate that miR-421 could directly target PINK1, thereby affecting mitochondrial function [24]. Our study showed that PINK1 expression was significantly downregulated in both PD cells and animal models. Moreover, a targeted binding site between miR-421 and PINK1 was also found, and it was proven that miR-421 could inhibit the occurrence of mitochondrial autophagy in PD by regulating the expression of PINK1.

In summary, our current studies demonstrated the function and molecular mechanism of miR-421 in PD development. Our results provide key therapeutic implications for PD treatment.

## Figures and Tables

**Figure 1:** miR-421 is highly expressed in SH-SY5Y cells and inhibits mitophagy. (a) The expression of miR-421 was detected by RT–qPCR. (b) The expression of miR-421 was detected by RT–qPCR. (c) The expression of apoptosis-related proteins was detected by Western blotting. (d) Apoptosis of cells was measured by flow cytometry. (e) The expression of LC3II/I was detected by Western blotting. (f) ROS generation was measured by ELISA. (g) Mitochondrial membrane potential was measured by flow cytometry. ∗*P* < 0.05, ∗∗*P* < 0.01, ∗∗∗*P* < 0.001.

**Figure 2:** MiR-421 targets PINK1. (a) Prediction of miR-421 and PINK1 targeted binding sites and dual-luciferase reporter assay. (b) The expression of PINK1 and Parkin was detected by Western blotting. ∗*P* < 0.05, ∗∗*P* < 0.01.

**Figure 3:** MiR-421 inhibits cell mitophagy via PINK1/Parkin. (a) Western blotting was used to detect the expression of PINK1 and Parkin. (b) The expression of Bax was detected by Western blotting. (c) Apoptosis of SH-SY5Y cells was detected by flow cytometry. (d) The expression of LC3II/I was detected by Western blotting. (e) ROS generation was measured by ELISA. (f) Mitochondrial membrane potential was measured by flow cytometry. ∗*P* < 0.05, ∗∗*P* < 0.01, ∗∗∗*P* < 0.001.

**Figure 4:** Inhibition of miR-421 attenuates neurodegeneration in mice. (a) The expression of miR-421 was detected by RT–qPCR. (b) The expression of PINK1 and Parkin was detected by Western blotting. (c) TH-positive neurons were analyzed by immunohistochemistry. ∗*P* < 0.05, ∗∗*P* < 0.01.

## Data Availability

The datasets used and/or analyzed during the current study are available from the corresponding author upon reasonable request.
